The article "Dissection of soybean populations according to selection signatures based on whole-genome sequences" was retracted in 2021. Reasons: an official misconduct investigation; misconduct by an author; concerns about the data.

# Dissection of soybean populations according to selection signatures based on whole-genome sequences

**DOI:** 10.1093/gigascience/giz151

**Published:** 2019-12-23

**Authors:** Jae-Yoon Kim, Seongmun Jeong, Kyoung Hyoun Kim, Won-Jun Lim, Ho-Yeon Lee, Namhee Jeong, Jung-Kyung Moon, Namshin Kim

**Affiliations:** 1 Genome Editing Research Center, Korea Research Institute of Bioscience and Biotechnology (KRIBB), Gwahak-ro 125, Yuseong-gu, Daejeon 34141, Republic of Korea; 2 Department of Bioinformatics, KRIBB School of Bioscience, University of Science and Technology (UST), Gajeong-ro 217, Yuseong-gu, Daejeon 34141, Republic of Korea; 3 National Institute of Crop Science, Rural Development Administration, Nongsaengmyeong-ro 370, Deokjin-gu, Jeon-Ju 54874, Republic of Korea

**Keywords:** *Glycine max*, soybean, population genetics, selection signature, whole-genome

## Abstract

**Background:**

Domestication and improvement processes, accompanied by selections and adaptations, have generated genome-wide divergence and stratification in soybean populations. Simultaneously, soybean populations, which comprise diverse subpopulations, have developed their own adaptive characteristics enhancing fitness, resistance, agronomic traits, and morphological features. The genetic traits underlying these characteristics play a fundamental role in improving other soybean populations.

**Results:**

This study focused on identifying the selection signatures and adaptive characteristics in soybean populations. A core set of 245 accessions (112 wild-type, 79 landrace, and 54 improvement soybeans) selected from 4,234 soybean accessions was re-sequenced. Their genomic architectures were examined according to the domestication and improvement, and accessions were then classified into 3 wild-type, 2 landrace, and 2 improvement subgroups based on various population analyses. Selection and gene set enrichment analyses revealed that the landrace subgroups have selection signals for soybean-cyst nematode HG type 0 and seed development with germination, and that the improvement subgroups have selection signals for plant development with viability and seed development with embryo development, respectively. The adaptive characteristic for soybean-cyst nematode was partially underpinned by multiple resistance accessions, and the characteristics related to seed development were supported by our phenotypic findings for seed weights. Furthermore, their adaptive characteristics were also confirmed as genome-based evidence, and unique genomic regions that exhibit distinct selection and selective sweep patterns were revealed for 13 candidate genes.

**Conclusions:**

Although our findings require further biological validation, they provide valuable information about soybean breeding strategies and present new options for breeders seeking donor lines to improve soybean populations.

The article "Dissection of soybean populations according to selection signatures based on whole-genome sequences" was retracted in 2021. Reasons: an official misconduct investigation; misconduct by an author; concerns about the data.

## Background

Soybean (*Glycine max* L. Merr.), one of the most economically important leguminous crops, originated from its annual wild relative *Glycine soja* (Sieb. and Zucc.) in China ∼5000 BC [1, 2]. Soybeans were first cultivated in earnest by ancient Chinese farmers ∼3000–1000 BC [3] and then spread to neighboring regions, Korea, and Japan, around the first century AD [4]. They were localized into a multitude of soybean landraces during this period [5, 6] and subsequently spread to North America around the 18th century AD [7, 8]. As molecular biology theories and biotechnologies were introduced into crop breeding programs from the 19th century onwards [9], modern breeders began to improve the soybean landraces in various ways. Since then, numerous improved soybean varieties have been developed, fulfilling diverse agronomic needs [10]. Currently, >170,000 landrace and improved soybean accessions in >70 countries are contributing to human and livestock as a major source of vegetable oil and protein [11].

Landrace populations have unique adaptive characteristics with considerable local diversity [12]. During domestication and subsequent geographical dispersion, landrace soybeans have spread to diverse environments, including cold/hot climates, humid/dry climates, and fertile plains to mountainous regions [13]. They have adapted successfully to these diverse environments by accumulating multiple genetic variations in all traits [14] and by developing the capacity to stabilize yields, increase fitness, and tolerate biotic and abiotic stress [6, 15]. For instance, PI 594527 and PI 567139B were reported to have excellent resistance to nearly all *Phytophthora sojae* races [16, 17], and PI 88788 was reported to possess resistance to most soybean-cyst nematode (SCN) *Heterodera glycines* (HG) races [18]. These characteristics have played a fundamental role in improving other populations, and many soybean breeders have developed a variety of improvement soybeans with distinct adaptive characteristics, based on the landrace's useful genetic materials [19]. For example, Keunolkong (developed from landraces in Kyungbuk province in Korea) was reported to have a large seed size with high yield, together with tolerance to lodging stress [20]. Also, PI 438471 (Fiskeby III), which was developed by crossing several accessions including landrace PI 548379, was reported to have high or partial tolerance to multiple abiotic stresses, including drought, salt, aluminum toxicity, iron deficiency, and atmospheric ozone pollution [21–23].

The article "Dissection of soybean populations according to selection signatures based on whole-genome sequences" was retracted in 2021. Reasons: an official misconduct investigation; misconduct by an author; concerns about the data.

Previous studies to date have focused on identifying genetic changes and selection signature differences between landrace and improvement soybeans. In terms of genetic diversity, Hyten et al. and Grainger et al. reported that landrace soybeans lost approximately half of their diversity due to domestication, and the improvement soybeans lost ∼28% more diversity through subsequent improvements [24, 25]. Concerning morphological features, Wen et al. reported that the small black seeds of the wild type (WT) changed to larger seeds of variable color (landrace soybean) and to much larger yellow seeds (improvement soybean) through successive rounds of positive selection [26]. In addition, Zhou et al. reported differences in selection signals for the oil content of seeds, with identifying 53 domesticated-selective sweep regions and 43 improvement-selective sweep regions [8]. These studies identified genetic variations of various agronomic traits and provided a genomic basis for improving soybean populations; however, they were limited with regard to revealing the genomic architectures of soybean subpopulations that adapted to diverse environments and multiple selection events [8, 24].

At the population level, a variety of selections and environmental pressures have generated genome-wide divergence within crop populations [27]. Previous studies demonstrated diverse population structures in soybean population and indicated the presence of their subpopulations: Valliyodan et al., on genomic diversity of 106 soybean whole genomes [28]; Zhou et al., on domestication and improvement signals in 302 soybean whole genomes [8]; Wen et al., on selection signatures in 1,404 soybean SoySNP50K chip datasets [26]; and Bandillo et al., on local adaptations in 3,012 soybean SoySNP50K chip datasets [6]. In the wider soybean population, these subpopulations also harbor their own selection signatures that could be utilized in soybean breeding programs [8]. Thus, research on identifying their adaptive characteristics and the genes controlling them is needed.

In this study, we re-sequenced a core set of 245 soybean accessions comprising 112 WT, 79 landrace, and 54 improvement soybeans, which were selected from 4,234 soybean accessions that our team generated previously using the 180 K Axiom® SoyaSNP array [29]. The aims of the study were as follows: (i) to identify the genomic architectures of WT, landrace, and improvement soybeans; (ii) to reveal their subpopulation structure; and (iii) to present selection signatures of the subpopulations together with candidate genes.

## Analyses

### Sample preparation and re-sequencing

A core set of 245 soybean accessions was selected for re-sequencing from a larger collection 4,234 accessions (see Methods). The core set covered 95% of the genotype diversity and frequency of the larger collection (Supplementary Fig. S1a and b) and comprised 112 WT and 133 cultivar-type (CT) soybeans, of which 54 were improved cultivar (IC) and 79 were landrace cultivar (LR) soybeans. The accessions originated in 8 countries: China, Japan, Korea, Russia, Canada, Sweden, Taiwan, and the USA. Korean accessions accounted for 67%, 87% and 81% of WT, IC, and LR accessions, respectively (Fig. 1A and Supplementary Table S1). In total, 31.3 billion reads of 97–151 bp (4.35 Tb of sequence) were generated and aligned to the soybean reference genome, Williams 82 assembly 2 annotation version 1 (Wm82.a2.v1) [30]. The average alignment rate was 98.12%, covering 96.85% of the reference genome, and the average read depth after removal of PCR duplicates was 16.38× (Additional File 2). A variant-calling process detected 35,812,378 raw variants, and 2,661,910 insertion/deletion polymorphism (indel) and 19,853,829 bi-allelic single-nucleotide polymorphism (SNP) variants were separated after quality-filtering processes (see Methods). Then, 9,650,073 bi-allelic SNPs with a minor allele frequency (MAF) of >1% were finally obtained from the entire 245 soybean accessions (Supplementary Table S2). This number of bi-allelic SNPs was similar to those reported by Zhou et al. (9,790,744) [8] and Valliyodan et al. (10,417,285) [28], which are previous studies on the whole genome of WT and CT soybeans. To further identify the variant distribution of each group, the variant-calling process was conducted for the WT, LR, and IC groups, in the same way (Supplementary Table S3). The number of bi-allelic SNPs was the highest for the WT group (15,933,086), followed by the LR (4,834,812) and IC (3,793,575) groups (Fig. 1B). The highest number of bi-allelic SNPs with a MAF of >1% was found in the WT group (10,426,662), followed by the LR (4,614,302) and IC (3,703,778) groups. The WT group also exhibited the highest number of missense SNPs with a MAF of >1% (420,582), followed by the LR (199,265) and IC (159,665) groups (Supplementary Table S4). In terms of bi-allelic SNP variants, the WT group had the largest number of variants, with numerous rare variants (5,506,424, MAF < 1%). The LR group had ∼69% fewer variants (11,098,274) than the WT group, due to the domestication process, and in particular, showed a considerable loss in rare variants (5,285,914). Due to the impact of the improvement process after domestication, the IC group had ∼21% fewer variants (1,041,237) than the LR group, and exhibited the smallest number of variants including functional variants such as missense. The variant loss rates of the LR and IC groups indicated that the impact on the allelic structures of variants was stronger in the domestication process than in the improvement process. From subsequent analyses, we used the 9,650,073 bi-allelic SNPs (MAF > 1%), which covers the entire 245 soybean accessions, except when examining the genomic measures of each group for genomic diversity (π), inbreeding coefficient (F), and linkage disequilibrium (LD). These measures were obtained from the bi-allelic SNPs (MAF > 1%) of each group (Supplementary Table S5).

The article "Dissection of soybean populations according to selection signatures based on whole-genome sequences" was retracted in 2021. Reasons: an official misconduct investigation; misconduct by an author; concerns about the data.

**Figure 1:** The numbers of accessions and bi-allelic SNPs for each group and subgroup. **A**, Distribution of accessions according to origin in each group (see Supplementary Table S1). **B**, Distribution of bi-allelic SNPs for each group. The x-axis indicates the number of bi-allelic SNPs concerning the reference genome (Wm82.a2.v1). The upper and lower bar plots of each group show the numbers of all bi-allelic SNPs and the bi-allelic SNPs filtered with MAF of < 1%, respectively (see Supplementary Table S3).

### Genomic architecture of WT and CT soybean groups

Severe genetic bottlenecks had occurred during the soybean domestication period and have considerably affected a loss of genetic diversity in the LR and subsequent IC [24]. In the core 245 accessions tested, π was highest for WT (1.69 × 10^−3^) and decreased to LR (0.96 × 10^−3^) and to IC (0.83 × 10^−3^) (Supplementary Table S5). The LR group lost ∼43% of π compared with the WT group, and the IC group lost ∼14% of π compared with the LR group. The large loss rate observed in the LR group, as compared to the IC group, was similar to the results reported in previous studies [8, 26, 31]. These results indicated that the domestication event had a marked effect on the allelic structure and that the later improvement process has influenced the narrow genomic regions encoding the traits of interest. As another measure of genomic architecture, LD level reflects various evolutionary pressures, including genetic bottlenecks and selection pressures [32, 33]. The average LD values within 500 kb were highest for the IC (0.2624), followed by LR (0.2011) and WT (0.0394) (Supplementary Table S5 and Fig. S2). This LD result well explained the LR's domestication event accompanied by conscious and unconscious selections, and the IC's improvement event accompanied by intensive conscious selections. The F, a measure of heterozygosity, was 0.9231, 0.8961, and 0.8982 for WT, LR, and IC, respectively (Supplementary Table S5). Although there were some differences among the 3 groups, all showed high F values due to their characteristics of stringent cleistogamy and inbreeding [15].

The article "Dissection of soybean populations according to selection signatures based on whole-genome sequences" was retracted in 2021. Reasons: an official misconduct investigation; misconduct by an author; concerns about the data.

### Population structure and relationship of WT and CT soybean groups

Multiple independent selections and diverse environmental pressures can lead to genome-wide divergence in a crop population [27]. Therefore, we examined the population structures and relationships between the WT, LR, and IC groups. Based on extensive population analyses, we classified WT, LR, and IC into 3 WT (WT-1, WT-2, and WT-3), 2 LR (LR-1 and LR-2), and 2 IC (IC-1 and IC-2) subgroups (Fig. 2). The WT subgroups were clustered according to their origins (China, Korea, and Japan, respectively) within a common large clade in the phylogenetic tree (Fig. 2A). They showed their own unique genomic compositions in structure analysis (Fig. 2B) and were clearly distinguished by the first and second principal components (PCs) in PC analysis (Fig. 2C). Their π decreased in the order of WT-1 (China origin), WT-2 (Korea origin), and WT-3 (Japan origin), with 1.88 × 10^−3^, 1.53 × 10^−3^, and 1.50 × 10^−3^ (Supplementary Table S5). This decreasing tendency, together with the phylogenetic and LD patterns (Fig. 2E), supports the hypothesis that all domesticated soybeans originated from 1 single domestication event in the China region [34]. In the LR group, LR-1 and LR-2 showed different genomic compositions and distinct clades (Fig. 2A and B). The 2 subgroups were clearly separated by the first PC, which explains ∼70.63% of the total genetic variation (Fig. 2D). Unlike the LR group, the IC-1 and IC-2 subgroups showed relatively similar genomic compositions on structure analysis (Fig. 2B). However, they had their own unique clade (Fig. 2A) and were separated by the second PC, which explains ∼8.65% of the total genetic variation (Fig. 2D and Supplementary Fig. S3). Also, they were genetically distinguished from each other, with a fixation index value (Fst) of 0.1067 (Supplementary Table S6).

**Figure 2:** Genomic relationship between IC, LR, and WT, including their subgroups. **A**, Phylogenetic tree inferred by the randomized and accelerated maximum likelihood method based on sequence alignments of all accessions. **B**, Population structure calculated by the maximum likelihood–based clustering algorithm. **C, D**, PC analysis plots for all groups and cultivar groups, calculated on the basis of genetic diversity. E, The extent of LD decay calculated up to 500 kb. **F**, Maximum likelihood tree for the relationships of the gene flow and genetic drift between the subgroups. The x-axis indicates the strength of genetic drift. The 3 arrows show the gene flows and migration rates derived from source groups, and the scale bar represents the standard error. The whole WT group was used as 1 root group in order to focus more on interactions among IC and LR subgroups while minimizing the standard error.

The article "Dissection of soybean populations according to selection signatures based on whole-genome sequences" was retracted in 2021. Reasons: an official misconduct investigation; misconduct by an author; concerns about the data.

The Fst statistic, which was calculated in a pairwise manner, confirmed that all subgroup pairs show high levels of genetic differentiation (>0.05); the exception was the IC-2 and LR-2 pair (Table S6). The IC-2 and LR-2 pair showed an Fst value of 0.0349, which is small enough to be considered as a single group. Structure analysis revealed a nearly identical genomic composition (Fig. 2B), and PC analysis revealed that they almost formed a single cluster (Fig. 2D). In addition, phylogenetic analysis showed that some of their accessions were mixed into each other's clades (Fig. 2A). When considering their different LD and genetic drift patterns (Fig. 2E and F), these similar genomic architectures indicated that the IC-2 subgroup was improved based mainly on the LR-2 subgroup, and that it has developed its own genome while maintaining a substantial portion of the genomic characteristics of LR-2.

The degree of gene flow and genetic drift among subgroups was further examined (Fig. 2F and Supplementary Fig. S4). The LR subgroups showed higher levels of genetic drift and higher LD values than the WT group due to the domestication process (Fig. 2E and F). The IC subgroups showed much higher values than the LR subgroups due to the subsequent improvement process. In this analysis, we found interaction signals between the WT, LR-1, and IC-1 subgroups (Fig. 2F). Approximately 34.7% of the IC-1 genome was derived from that of LR-1, and 36.7% of the LR-1 genome was derived from that of WT. Notably, the IC-1 subgroup was differentiated directly from LR-2 and later IC-2, and showed the highest genetic drift and LD values (Fig. 2E and F). These results indicated that the LR-1 subgroup has conserved a substantial proportion of the genomic characteristics derived from the WT group (Fig. 2B), and that the IC-1 subgroup has formed its own genomic characteristics through extensive improvements based on various groups.

### Detection of selection signals in CT soybean subgroups

Crop domestication and improvement involves unconscious and conscious selections [26], and these processes select favorable alleles associated with beneficial traits that enhance the crops' fitness, agronomic features, morphological features, or biotic and abiotic tolerance [35]. Many crop populations developed by farmers or breeders have these traits as adaptive characteristics, and these characteristics are utilized as invaluable genetic materials for improving other populations in various breeding programs [19, 24]. With this in mind, we performed a pairwise comparison of the IC-1, IC-2, LR-1, and LR-2 genomes to identify their selection signatures. The cross-population composite likelihood ratio (XP-CLR) [36] method was used to examine genomic regions in which allele frequencies were highly differentiated. This XP-CLR method is more robust to ascertainment bias of SNP discovery than allele frequency spectrum–based methods, and it provides more statistical power than the CLR, Fst, and Tajima D methods [36, 37]. Additionally, this method was adopted widely by previous studies to detect selective sweep regions in crops such as soybean [8, 26], wheat [27], upland cotton [38], and rice [39]. After the calculation, a strict cut-off line was set to exclude as many false-positive regions as possible. Outlier regions belonging to the top 1% of the empirical distributions of the XP-CLR statistic were considered as candidate selected regions (Supplementary Figs S5 and S6a–l), and genes within these regions were designated as candidate selected genes (Additional File 3). Next, we examined common candidate genes for each subgroup, which exhibited common selection signals against all of the other 3 subgroups. Although 1 subgroup may have various adaptive characteristics against each of the other subgroups, we focused on identifying unique adaptive characteristics that 1 subgroup has in common for all 3 remaining subgroups, in accordance with our goal of presenting useful subgroups that can be utilized and referenced in future breeding studies and programs. Moreover, this approach using common candidate genes was able to reduce some false-positive results in identifying adaptive characteristics of each subgroup because our subgroups classified by genomic similarity might contain a little variability for the group classification. Therefore, we extracted common candidate genes for each subgroup and considered these genes as a gene set representing each subgroup. The numbers of candidate genes in the gene sets of IC-1, IC-2, LR-1, and LR-2 were 422, 235, 454, and 258, respectively (Supplementary Fig. S7a–d). A gene set enrichment analysis (GSEA) was then performed for the 4 gene sets, and 67, 107, 112, and 87 Gene Ontology (GO) terms of raw *P*-value < 0.05 were obtained in IC-1, IC-2, LR-1, and LR-2, respectively (Additional File 4). The non-adjusted *P*-value was used to broadly capture relationships between the GO terms. To confirm the selection signals in which the GO terms are commonly involved, a hierarchical relationship analysis between GO terms was conducted using the QuickGo web-based tool [40], and then 2, 1, 3, and 3 hierarchical relationship trees containing the top 10% of GO terms by raw *P*-value were detected in IC-1, IC-2, LR-1, and LR-2 (Supplementary Figs S8–S11). On the basis of major GO terms that are the sources of the hierarchical relationship trees, we revealed selection signals for each subgroup: IC-1 was plant growth, development, and viability; IC-2 was seed development with embryo development; LR-1 was defense responses to SCN HG type 0; and LR-2 was seed development with germination (Table 1). Including both the GO terms identified in the relationship trees and those reported in previous studies, the total numbers of GO terms involved in the selection signals were 34, 45, 62, and 43 in IC-1, IC-2, LR-1, and LR-2, respectively. The GO terms are summarized with references in Additional File 4, and 5 representative GO terms with major GO terms are provided in Table 1.

The article "Dissection of soybean populations according to selection signatures based on whole-genome sequences" was retracted in 2021. Reasons: an official misconduct investigation; misconduct by an author; concerns about the data.

**Table 1:** Selection signatures and 5 representative GO terms identified in GSEA (see Additional File 4 for all significant GO terms)

Group	No. of GO terms^a^	No. of genes^b^	Representative GO terms^c^		Gene count	Raw *P*-value	Rank of *P*-value^d^	Association^e^	Reference^f^
**Plant growth, development, and viability**									
IC-1	34 (67)	83 (115)	GO:0050896	Response to stimulus	42	2.10E−12	1	Brassinosteroid transcription factor	[52]
			GO:0016128	Phytosteroid metabolic process	7	2.26E−08	3	Plant growth and development	[53]
			*GO:0042742	Defense response to bacterium	8	6.35E−07	4	Plant viability	[54, 55]
			GO:0042446	Hormone biosynthetic process	6	5.88E−05	18	Plant growth and development	[56]
			*GO:0016132	Brassinosteroid biosynthetic process	3	1.04E−03	26	Plant growth, development, and immunity	[53, 57, 58]
**Seed and embryo development**									
IC-2	45 (107)	84 (88)	GO:0010154	Fruit development	14	3.51E−23	6	Seed development	[59, 60]
			GO:0048316	Seed development	12	7.78E−20	7	Seed development and maturation	[61, 59, 62]
			GO:0032012	Regulation of ARF protein signal transduction	4	1.44E−10	16	Seed development and yield	[63, 64]
			*GO:0009793	Embryo development ending in seed dormancy	6	5.04E−10	19	Seed development and maturation	[61, 62, 65]
			GO:0009790	Embryo development	5	5.39E−10	20	Seed development, size, and yield	[66–70]
**Defense response to SCN HG type 0**									
LR-1	62 (112)	203 (204)	GO:0051707	Response to other organism	15	5.75E−15	3	Resistance to SCN HG type 0	[71]
			GO:0006952	Defense response	10	2.26E−09	8	Resistance to SCN HG type 0	[72, 73]
			*GO:0045087	Innate immune response	6	3.88E−06	20	Resistance to SCN HG type 0, 2, 5, 7	[72, 74]
			*GO:0009624	Response to nematode	1	7.95E−03	74	Resistance to SCN HG type 0	[75, 76]
			*GO:0051172	Negative regulation of nitrogen compound metabolic process	8	8.52E−03	75	Resistance to SCN HG type 0	[72]
**Seed development and germination**									
LR-2	43 (87)	118 (119)	GO:0010154	Fruit development	9	2.68E−13	2	Seed development	[59, 60]
			GO:0048316	Seed development	8	6.06E−12	4	Seed development and maturation	[61, 59, 62]
			*GO:0043043	Peptide biosynthetic process	5	2.48E−10	12	Seed germination	[77, 78]
			*GO:0010029	Regulation of seed germination	3	3.22E−06	26	Seed germination	[79]
			*GO:0010431	Seed maturation	2	4.05E−05	42	Seed development and maturation	[59]

a The number of GO terms associated with selection signature. Parenthesis indicates the total number of significant GO terms.

b The number of candidate genes enriched in GO terms related to selection signature. Parenthesis indicates the total number of candidate genes identified in all significant GO terms.

c The 5 representative GO terms related to selective signature. Major GO terms identified in the hierarchical relationship trees (Supplementary Figs S8–S11) are marked with an asterisk. All GO terms are summarized in Additional File 4.

d Rank of the corresponding GO term in ascending order of raw *P*-values of all significant GO terms.

e Description of GO term reported related to selection signature.

f References to the description in the “Association” column. ARF: auxin response factor.

The article "Dissection of soybean populations according to selection signatures based on whole-genome sequences" was retracted in 2021. Reasons: an official misconduct investigation; misconduct by an author; concerns about the data.

At the genome level, selection processes leave detectable traces in patterns of nucleotide diversity, LD, and allele frequency because they change the neutral pattern of the genome under the neutral theory of molecular evolution [41]. Generally, nucleotide diversity and haplotype diversity decrease, and LD increases, under directional selection [42]. Also, according to the hitchhiking theory, alleles of closely linked loci are affected when an allele of a specific locus is affected by selection [43, 44]. This process, termed selective sweep, characteristically leaves long-range haplotypes with low diversity [45]. Therefore, to clarify the selection signatures of each subgroup, we examined the genomic patterns of candidate genes belonging to the top 0.5% of the empirical distributions of the XP-CLR statistic in gene sets of each subgroup (Figs 3, 4, and Supplementary Fig. S6a−l). The patterns of nucleotide diversity, haplotype diversity, and LD were investigated using the methods presented by Hudson et al. [46], Nei [47], and Kelly [48], respectively (Figs 3A and B and 4A and B). The hitchhiking process was examined for regions containing missense variants and their surrounding 14 variants, and was identified through the haplotype structures and frequencies of the regions (Figs 3C and D, 4C and D, and Additional File 5). In addition, the long-range haplotype was confirmed using the haplotype-sharing degree approach that indirectly presents extended-haplotype regions by visualizing the minor and major alleles of each variant as red and yellow (Figs 3A and B and 4A and B). In the plot for the degree of haplotype sharing, wider area of variants that do not mix vertically with other colors indicates that a subgroup has a longer-range haplotype and lower haplotype diversity for the area. This haplotype-sharing degree approach was used similarly in several other studies related to selection analysis [49–51]. Through these analyses, we detected 13 candidate genes that have distinctive selection patterns along the selection signals of each subgroup (Table 2).

The article "Dissection of soybean populations according to selection signatures based on whole-genome sequences" was retracted in 2021. Reasons: an official misconduct investigation; misconduct by an author; concerns about the data.

**Figure 3:** Selection signatures for the IC-1 and IC-2 subgroups. **A, B**, Patterns of nucleotide diversity, haplotype diversity, and linkage disequilibrium (*top*) and the degree of haplotype sharing among all subgroups (*bottom)* in Glyma.16g210300 and Glyma.03g144400. The Glyma.16g210300 and Glyma.03g144400 genes are located at 36,943,073–36,948,828 bp on chromosome 16 and at 36,004,707–36,005,955 bp on chromosome 3, respectively. All 7 subgroup lines are shown for the nucleotide and haplotype diversities. For clarity of the subgroup lines, only the IC-1 and IC-2 subgroup lines are shown for the linkage disequilibrium. Detailed illustrations of the 3 patterns are provided in Supplementary Figs S12a–c and S14a–c. The plots for the degree of haplotype sharing are displayed for all variants in the entire regions of 2 genes, and the major and minor alleles of each variant are presented in red and yellow, respectively. **C, D**, Gene structures and haplotype frequencies for regions containing 1 missense variant in Glyma.08g323200 and Glyma.03g022900, respectively. The gene structures are displayed on the top, and regions containing the missense variant and its surrounding 14 variants are drawn beneath them. Reference and alternative alleles (Allele 1 and 2) are presented in green and yellow, and missense variants are highlighted in light yellow. The missense variants of the Glyma.08g323200 and Glyma.03g022900 genes are located at 44,174,550 bp on chromosome 8 (p.Pro191Arg on rs388102659) and at 2,415,948 bp on chromosome 3 (p.Arg560His on rs392782287), respectively. The haplotype structures for those regions are depicted below the gene structures, with haplotype frequencies shown to the right. Only the top 2 haplotype frequencies are displayed for each subgroup owing to illustration constraints. Information regarding all haplotype frequencies is provided in Additional File 5.

**Figure 4:** Selection signatures for the LR-1 and LR-2 subgroups. **A, B**, Patterns of the nucleotide diversity, haplotype diversity, and linkage disequilibrium (*top*) and the degree of haplotype sharing among all subgroups (*bottom*) in Glyma.03g051100 and Glyma.12g181400. The Glyma.03g051100 and Glyma.12g181400 genes are located at 6,684,296–6,686,809 bp on chromosome 3 and at 34,193,664–34,197,110 bp on chromosome 12, respectively. All 7 subgroup lines are shown for the nucleotide and haplotype diversities. For clarity of the subgroup lines, only the LR-1 and LR-2 subgroup lines are shown for the linkage disequilibrium. Detailed illustrations of the 3 patterns are provided in Supplementary Figs S16a–c and S18a–c. The plots for the degree of haplotype sharing are shown for all variants in the entire regions of 2 genes, and the major and minor alleles of each variant are marked red and yellow, respectively. **C, D**, Gene structures and haplotype frequencies for regions containing 2 and 1 missense variants in Glyma.06g316300 and Glyma.13g369100, respectively. The gene structures are illustrated on the top, and regions containing the missense variant and its surrounding 14 variants are shown beneath them. Reference and alternative alleles (Alleles 1 and 2) are marked green and yellow, and missense variants are highlighted in light yellow. The missense variants of the Glyma.06g316300 and Glyma.13g369100 genes are located at 50,518,313 and 50,518,392 bp on chromosome 6 (p.Ile34Thr on rs123802993 and p.Phe8Ile on rs123802994) and at 45,466,067 bp on chromosome 13 (p.Thr218Ile on rs125880759), respectively. The haplotype structures for those regions are depicted below the gene structures, with haplotype frequencies shown to the right. Only the top 2 haplotype frequencies are displayed for each subgroup due to illustration constraints. Information regarding all haplotype frequencies is provided in Additional File 5.

The article "Dissection of soybean populations according to selection signatures based on whole-genome sequences" was retracted in 2021. Reasons: an official misconduct investigation; misconduct by an author; concerns about the data.

**Table 2.** Genes with unique selection patterns among candidate genes enriched significantly in GO terms (see Additional File 4 for all candidate genes enriched in the GO terms)

Group	Candidate gene^a^	*Arabidopsis* gene^b^	XP-CLR score range^c^	Associated GO IDs^d^	Reference^e^
**Plant growth, development, and viability**					
IC-1	Glyma.08G323200	AT3G07040	(5.15, 7.78)	GO:0006952	[82]
	Glyma.16G170700	AT2G34930	(9.01, 20.34)	GO:0006950, GO:0050896	[83]
	Glyma.16G210300	AT1G73340	(3.01, 5.55)	GO:0006694, GO:0007275, GO:0009058, GO:0010817, GO:0016125, GO:0016128, GO:0016129, GO:0016131, GO:0016132, GO:0032501, GO:0042446, GO:0055088, GO:1901362, GO:1901576, GO:1901615, GO:1901617	[84]
	Glyma.18G226500	AT4G26090	(36.12, 108.19)	GO:0006952	[85]
**Seed and embryo development**					
IC-2	Glyma.03G022900	AT3G60860	(4.45, 9.43)	GO:0032012	[86]
	Glyma.03G144400	AT5G06760	(2.92, 5.72)	GO:0009793	[87]
**Defense response to SCN HG type 0**					
LR-1	Glyma.03G051100	AT5G01550	(2.99, 6.22)	GO:0009607, GO:0009617, GO:0042742, GO:0043207, GO:0050896, GO:0051707	[71]
	Glyma.06G316300	AT3G07040	(3.62, 6.21)	GO:0006952, GO:0007165	[88]
	Glyma.14G047900	AT4G08850	(2.97, 6.11)	GO:0016310	[89–91]
**Seed development and germination**					
LR-2	Glyma.12G028300	AT3G19820	(5.14, 7.26)	GO:0008152, GO:0008202, GO:0048367, GO:0071704	[92]
	Glyma.12G028400	AT3G18630	(5.14, 7.26)	GO:0009987	[92]
	Glyma.12G181400	AT5G03740	(4.68, 7.01)	GO:0007275, GO:0008152, GO:0010154, GO:0032501, GO:0048316, GO:0048608, GO:0048731, GO:0061458, GO:0071704	[93, 94]
	Glyma.13G369100	AT1G80640	(5.90, 6.44)	GO:0006468	[95]

a Candidate gene associated with selection signature, belonging to the top 0.5% of the empirical distributions of XP-CLR results.

b Best-hit *Arabidopsis* gene name, corresponding to the soybean gene.

c Range of minimum and maximum values of normalized XP-CLR scores for the other 3 subgroups. All XP-CLR results are summarized in Additional File 3.

d GO IDs associated with the candidate gene in our results.

e References to the candidate gene reported related to selection signature.

### Adaptation of IC-1 to plant growth, development, and viability

Plant sterols and steroid hormones, brassinosteroids (BRs), and their precursors, phytosterols, are compounds affecting a wide range of biological activities throughout the plant kingdom [53]. At the cellular level, BRs accelerate cell division, elongation, and differentiation [80], and at the organismal level, they regulate plant growth and development, flowering time, senescence, and various abiotic and biotic stresses [81]. The BRs have been reported to have a positive effect on plant growth and development in soybeans [57], as well as on fiber development in cotton [52]. Through the selection analysis comparing IC-1 with the other 3 subgroups, we revealed that IC-1 harbors selection signals on the BRs and defense signaling pathways involved in plant growth, development, and viability (Table 1 and Additional File 4).

A total of 67 GO terms were significantly enriched with 115 candidate genes. Of these, 34 GO terms with 83 candidate genes were associated with the BRs and defense response pathways (Table 1 and Additional File 4). Among these 34 GO terms, we found 2 major GO terms, GO:0016132 (Brassinosteroid biosynthetic process) and GO:0042742 (Defense response to bacterium), and also detected 15 and 8 other GO terms that are directly related to these 2 GO terms, respectively (Supplementary Fig. S8a and b). GO:0016132 was associated with the BR's biosynthesis, regulation, metabolism, and transport in plant organisms, together with 5 GO terms including GO:0016128 (Phytosteroid metabolic process) [53]. GO:0042742 was related to growth, development, and defense response of soybean, together with 3 GO terms [54]. In addition, GO:0050896 (Response to stimulus) was associated with the BRs and BR's transcription factor in cotton [52], and GO:0042446 (Hormone biosynthetic process) was related to growth and development in *Arabidopsis* [56] (Table 1).

The article "Dissection of soybean populations according to selection signatures based on whole-genome sequences" was retracted in 2021. Reasons: an official misconduct investigation; misconduct by an author; concerns about the data.

We further investigated Glyma.16g170700, Glyma.16g210300, and Glyma.18g226500 among the 83 candidate genes of the IC-1 subgroup (Table 2). Glyma.16g170700, an ortholog of the *Arabidopsis* AT2G34930 gene, encodes a disease resistance family protein [96] and has been identified as a candidate gene contributing to the plant immune system against pathogen infection in soybean [83]. Glyma.16g210300 (AT1G73340) encodes a cytochrome P450 superfamily protein and has been reported to be involved in the defense response to insects in *Arabidopsis* [84]. Glyma.18g226500 (AT4G26090) encodes an NB-ARC domain–containing disease resistance protein and has been reported as one of the disease resistance candidate genes in soybean [85]. In the entire regions of these 3 genes, the IC-1 subgroup showed the lowest nucleotide and haplotype diversity patterns and relatively long range of homogeneous haplotype patterns distinguished from the other subgroups (Fig. 3A and Supplementary Figs S12a–c and S13a–b). Also, as an indicator of strong selection, the IC-1 subgroup exhibited the highest LD values in regions around the 33.1011, 36.9467, and 51.5152 Mb positions of Glyma.16g170700, Glyma.16g210300, and Glyma.18g226500 genes, respectively. Additionally, another candidate gene, Glyma.08g323200 (AT3G07040), which encodes the same protein as Glyma.18g226500 and is related to immunity in *Arabidopsis* [82], exhibited a trace of the selective sweep with a missense variant (p.Pro191Arg) in the IC-1 subgroup (Fig. 3C). This variant was located at 44,174,550 bp position (rs388102659) and showed a tendency to have “G” allele type together with “A” allele type of a nearby variant (44,174,678 bp position). The haplotype frequencies of this region containing the 2 allele types were the highest for IC-1 (0.906), followed by IC-2, LR-1, WT-1, LR-2, WT-2, and WT-3 (0.091, 0.023, 0.021, 0, 0, and 0, respectively) (Additional File 5). Other subgroups, including WT subgroups, maintained this swept region at very low frequencies, but the IC-1 subgroup harbored this region at a high frequency along with the hitchhiking event.

### Adaptation of IC-2 and LR-2 to seed development

Seed weight (SW), one of the major yield components of soybean, influences the production of various soy foods such as edamame, natto, and nuts [97]. The SW trait is affected by various genetic and environmental factors during the seed development stage [98] and is also partially related to seed germination [99]. Before examining the adaptive characteristics of each subgroup, we determined 100-SW of each accession through phenotype survey, and compared mean and median values between subgroups using the Student *t*-test and Wilcoxon rank-sum test (Fig. 5). These 2 tests were used to indirectly refer to SW differences between the subgroups because their statistics might contain a bias due to small sample sizes of some subgroups. As a result of the 2 tests, we identified that the IC-2 and LR-2 subgroups show a tendency to have heavier 100-SW characteristics than the other 2 subgroups. Subsequently, through the selection analysis, we revealed that their heavy SW characteristics are associated, at least in part, with the adaptation process. The IC-2 and LR-2 subgroups exhibited selection signals on seed development in common (Table 1 and Additional File 4). As a slight difference, the IC-2 involved embryo development signals and the LR-2 accompanied seed germination signals.

The article "Dissection of soybean populations according to selection signatures based on whole-genome sequences" was retracted in 2021. Reasons: an official misconduct investigation; misconduct by an author; concerns about the data.

**Figure 5:** Box plot for 100-SW trait. The tables in this figure show *P*-values for 2-sample *t*-test (*left*) and Wilcoxon rank-sum test (*right*) calculated for all subgroup pairs. Top and bottom of the box indicate the interquartile range, and their whiskers mean 1.5 × interquartile range. Horizontal line and marker "X" indicate the median and mean values of accessions, and empty circles represent accessions observed outside the interquartile range (see Additional File 2 for phenotype information).

One hundred seven GO terms with 88 candidate genes were significantly enriched in the IC-2 subgroup. Of these, 45 GO terms with 84 candidate genes were associated with seed development (Table 1 and Additional File 4). Among the GO terms, GO:0009793 (Embryo development ending in seed) and GO:0048316 (Seed development) were involved in the final stage of seed maturation in *Arabidopsis* and *Medicago* [96, 61]; GO:0032013 (Regulation of ARF protein signal transduction) was related to seed development and weight in rapeseed [63]; GO:0010154 (Fruit development) was involved in pod maturity in soybean and *Medicago* [59, 60]; and GO:0009790 (Embryo development) was related to seed development, size, and yield in many plant organisms [66–70]. Particularly, GO:0009793 was detected alongside 14 directly related GO terms (Supplementary Fig. S9). Among the 84 candidate genes, we further identified Glyma.03g144400 (AT5G06760) and Glyma.03g022900 (AT3G60860) genes, which show unique selection patterns (Table 2). Glyma.03g144400 encodes a late-embryogenesis–abundant 4–5 protein and has been reported as a candidate gene associated with seed development in soybean [87]. Glyma.03g022900 encodes a SEC7-like guanine nucleotide exchange family protein and has also been reported as a candidate gene influencing seed yield in soybean [86]. As evidence of the selection process for Glyma.03g144400, the IC-2 subgroup showed the lowest nucleotide and haplotype diversity patterns and long-range homozygous haplotype patterns, together with the highest LD pattern (Fig. 3B and Supplementary Figs. S14a–c). In addition, for Glyma.03g022900, the IC-2 subgroup exhibited a fixed missense variant (p.Arg560His) at 2,415,948 bp (rs392782287) region showing a high LD value (Fig. 3D and Supplementary Fig. S15a–c). The haplotype frequencies of this region containing the missense variant were the highest for IC-2 (1.000), followed by LR-2, IC-1, WT-2, WT-3, LR-1, and WT-1 (0.605, 0.250, 0.096, 0.067, 0.045, and 0, respectively) (Additional File 5). Other subgroups retained this variant at low frequency in several haplotype structures, but the IC-2 subgroup possessed it in the completely fixed state in just 2 haplotype structures as a result of the selection process.

The article "Dissection of soybean populations according to selection signatures based on whole-genome sequences" was retracted in 2021. Reasons: an official misconduct investigation; misconduct by an author; concerns about the data.

In the LR-2 subgroup, 87 GO terms were significantly enriched with 119 candidate genes. Of these, 43 GO terms with 118 candidate genes were associated with seed development (Table 1 and Additional File 4). Three major GO terms, GO:0010431 (Seed maturation), GO:0010029 (Regulation of seed germination), and GO:0043043 (Peptide biosynthetic process) were identified along with 6, 10, and 6 directly related GO terms, and were related to seed development and germination in soybean, barley, and *Medicago* [59, 77–79] (Supplementary Fig. S11a–c). In addition, 4 GO terms were related to seed germination in soybean [77], 4 GO terms were associated with seed development and size in grape [70], and 2 GO terms (GO:0048316 and GO:0010154) were related to seed development as identified in the IC-2 subgroup (Additional File 4). Among their 118 candidate genes, we focused on Glyma.12g181400 (AT5G03740) and Glyma.13g369100 (AT1G80640) genes, which encode histone deacetylase 2C and kinase superfamily protein, respectively. Glyma.12g181400 has been reported as a candidate gene influencing seed development and germination in *Arabidopsis* [93, 94]. Due to the impact of the selection process, the LR-2 subgroup showed the lowest nucleotide and haplotype diversity patterns, high LD values, and relatively long-range haplotype than the other subgroups in this gene (Fig. 4A and Supplementary Fig. S16a–c). For Glyma.13g369100, which has been reported to be involved in embryo initiation of plant organisms [95], LR-2 exhibited a trace of selective sweep with a missense variant (p.Thr218Ile) (Fig. 4C). This variant was found at 45,466,067 bp position (rs125880759) and showed a tendency to have “T” allele type together with “T” and “T” allele types of 2 nearby variants (45,466,008 and 45,466,378 bp positions). The haplotype frequencies of this swept region were the highest for LR-2 (0.947) and the other subgroups maintained low/moderate frequencies (Additional File 5). In addition to these 2 genes, we also found 9 candidate genes belonging to quantitative trait loci (QTL) regions of soybean SW trait. Glyma.01g032900, Glyma.01g057100, Glyma.01g075000, Glyma.01g075100, and Glyma.01g075400 were involved in seed weight QTL 18–1.1 and Glyma.12g028200, Glyma.12g028300, Glyma.12g028400, and Glyma.12g028500 were involved in seed weight QTL 16–3, in the *G. max* v1.1 gene model [92]. Notably, for Glyma.12g028300 and Glyma.12g028400, we confirmed that the LR-2 subgroup exhibited long-range and low-diverse haplotype patterns with high LD values as a result of the selection process, with the exception of the region ∼2.1169 Mb in which haplotype diversity was the highest (Supplementary Fig. S17).

The article "Dissection of soybean populations according to selection signatures based on whole-genome sequences" was retracted in 2021. Reasons: an official misconduct investigation; misconduct by an author; concerns about the data.

### Adaptation of LR-1 to SCN HG type 0

The SCN, *Heterodera glycines* (HG), is one of the most destructive pests affecting seed yield in soybean. Many approaches have been proposed to control the SCN; of these, using resistant varieties has been suggested as an effective and practical method [100]. This approach is based mainly on 7 resistant varieties (Peking, PI 88788, PI 90763, PI 437654, PI 209332, PI 89772, and PI 548316) and uses a classification system that distinguishes these varieties into 8 types, numbered from 0 to 7, according to their vulnerability to SCN populations [101, 102]. This system is called the HG type system, where HG type 0 means that the SCN populations cannot reproduce >10% on all 7 varieties. In our study, the LR-1 subgroup contained all of these 7 varieties and showed selection signals for the SCN HG type 0 (Table 1 and Additional Files 1 and 4).

One hundred twelve GO terms with 204 candidate genes were enriched significantly; of these, 62 GO terms with 203 candidate genes were associated with resistance to SCN (Table 1 and Additional File 4). Three major GO terms, GO:0009624 (Response to nematode), GO:0045087 (Innate immune response), and GO:0051172 (Negative regulation of nitrogen compound metabolic process) were detected along with 6, 10, and 6 directly related GO terms (Supplementary Fig. S10a–c), and were related to SCN HG type 0, in common [72, 74–76]. In addition, 11 GO terms including GO:0051707 (Response to other organism) and GO:0006952 (Defense response) were related to resistance to SCN HG type 0 in soybean [71, 73], and 6 GO terms were related to resistance to SCN HG type 0 and type 1.2.5.7 in soybean [72, 103] (Additional File 4).

The article "Dissection of soybean populations according to selection signatures based on whole-genome sequences" was retracted in 2021. Reasons: an official misconduct investigation; misconduct by an author; concerns about the data.

We further examined Glyma.03g051100, Glyma06g316300, and Glyma.14g047900 among the 203 candidate genes (Table 2). Glyma.03g051100 (AT5G01550) encodes a lectin receptor kinase a4.1 protein and has been reported as a candidate gene involved in SCN type 0 resistance in soybean [71]; Glyma.14g047900 (AT4G08850), which encodes a leucine-rich repeat receptor-like protein kinase family protein, belongs to SCN QTL 3-g10 [96, 89] and has also been reported as one of the candidate genes involved in SCN type 0 and type 2.5.7 resistances in soybean [90, 91]. In the regions of these 2 genes, the LR-1 subgroup showed the lowest nucleotide and haplotype diversity patterns and long-range haplotypes distinguished from the other subgroups (Fig. 4B and Supplementary Figs S18a–c and S19). As traces of strong selection pressure, the LR-1 subgroup exhibited 3 high LD peaks at the 66,820, 66,860, and 66,870 Mb positions in Glyma.03g051100 (Fig. 4B) and a high LD region at 3.6703–3.6777 Mb in Glyma.14g047900 (Supplementary Fig. S19). Additionally, another candidate gene, Glyma.06G316300 (AT3G07040), which has been reported to be involved in plant defense signaling in *Arabidopsis* [88], exhibited a region affected by selective sweep in the LR-1 subgroup (Fig. 4D). This region had 2 missense variants positioned at 50,518,313 and 50,518,392 bp (rs123802993 and rs123802994), and the LR-1 showed a tendency to have “G” allele type at 50,518,313 bp and “T” allele type at 50,518,392 bp, simultaneously. The haplotype frequencies of this region containing the variants were the highest for LR-1 (0.932), followed by LR-2, IC-1, IC-2, WT-1, WT-2, and WT-3 (0.421, 0.318, 0.125, 0.125, 0.068, and 0.067, respectively) (Additional File 5). Other subgroups retained these 2 variants at low/moderate frequencies, whereas the LR-1 subgroup possessed them at a high frequency close to fixed variants as a result of the selection process.

## Discussion

### Genomic architecture of soybean subgroups

Domestication and geographical dispersion across diverse environments have generated a number of landrace soybeans with locally adapted characteristics, and modern breeding efforts based mainly on these landraces have developed a variety of improved soybeans with artificially adapted characteristics [104, 105]. These processes, accompanied by conscious and unconscious selections, have led to genome-wide divergence and stratification of the soybean population [8, 13]. Here, we analyzed the population structure of 245 soybean core accessions comprising 112 WT, 79 LR, and 54 IC accessions (Fig. 1A) and then classified them into 3 WT (WT-1, WT-2, and WT-3), 2 LR (LR-1 and LR-2), and 2 IC (IC-1 and IC-2) subgroups based on various population analyses. Each soybean subgroup was clustered according to genomic similarity and exhibited its own genomic architecture. The WT subgroups were clustered along their collection regions (Fig. 1A) and were sequentially differentiated in the order WT-1 (China), WT-2 (Korea), and WT-3 (Japan), indicating a single domestication event from the China region (Fig. 2A). The LR-1 subgroup showed a considerable genetic interaction with the WT group (Fig. 2F) and represented a distinct genomic structure with some similarity to WT genomic composition (Fig. 2A–E). The IC-1 subgroup exhibited a genomic architecture distinct from the other subgroups (Fig. 2D) and showed the highest levels of genetic drift and LD, suggesting strong selection pressure (Fig. 2E and F). The LR-2 and IC-2 subgroups showed similar genomic structures, differentiation levels, and heavy 100-SW characteristics, but they exhibited considerably different LD patterns, indicating differences in selection pressures (Figs 2B–E, 5, and Supplementary Table S6). These results suggest that different environmental pressures and conscious selections by farmers caused genomic divergence between LR-1 and LR-2, and subsequent conscious selections by breeders based on landrace induced genomic differences between IC-1 and IC-2. These results also suggest that the IC-2 subgroup has been improved for various agronomic purposes while maintaining SW characteristics derived mainly from the LR-2 subgroup. Additionally, these findings indicate that each subgroup may have unique adaptive characteristics, along with their own genomic architecture.

The article "Dissection of soybean populations according to selection signatures based on whole-genome sequences" was retracted in 2021. Reasons: an official misconduct investigation; misconduct by an author; concerns about the data.

### Adaptive characteristics of soybean subgroups

During environmental adaptations and artificial selections, soybean populations have developed their own adaptive characteristics enhancing their fitness, agronomic traits, morphological features, or tolerance for biotic and abiotic stresses. These characteristics and available germplasm sets provide an essential base as genetic materials and resources that can be used to improve other soybean populations [24]. From this perspective, we conducted extensive selection and gene set enrichment analyses and then revealed the selection signatures of 4 distinct soybean subgroups: LR-1's is resistance to SCN HG type 0; LR-2's is seed development with germination; IC-1's is plant growth, development, and viability; IC-2's is seed development with embryo development (Table 1 and Additional File 4). The LR-1 subgroup, which contains the 7 major accessions with resistance to various SCN races, showed selection signals for SCN HG type 0 (Table 1). The 62 GO terms were related to SCN responses, of which GO:0009624 (Response to nematode), GO:0045087 (Innate immune response), and GO:0051172 (Negative regulation of nitrogen compound metabolic process) were involved as major GO terms (Supplementary Fig. S10a–c). Among the 203 candidate genes enriched in the GO terms, Glyma.03g051100 and Glyma.14g047900 (belonging to the SCN 3-g10 QTL) genes exhibited the distinctive selection patterns (Table 2, Fig. 4B, and Supplementary Fig. S19) and Glyma.06g316300 exhibited the trace of selective sweep with 2 missense SNPs (Fig. 4D and Additional File 5). Both the LR-2 and IC-2 subgroups, which had significantly heavier 100-SW properties than the other subgroups (Fig. 5), showed selection signals associated with seeds. The LR-2 subgroup had 118 candidate genes with 43 GO terms related to seed development and germination (Table 1), some of which exhibited unique selection patterns and belonged to the seed weight QTLs, 18–1.1 and 16–3 (Fig. 4A and C). Similarly, the IC-2 subgroup had 84 candidate genes with 45 GO terms related to seed and embryo development (Table 1). Of these, Glyma.03g144400 (associated with seed development) showed distinct selection patterns with long-range haplotype patterns (Fig. 3B) and Glyma.03g022900 (associated with seed yield) exhibited 1 fixed missense SNP in a high LD peak (Table 2, Fig. 3D, and Supplementary Fig. S15c). In common, these 2 subgroups possessed both GO:0048316 (Seed development) and GO:0010154 (Fruit development) associated with seed development (Table 1 and Supplementary Figs S9 and S11a). The IC-1 subgroup showed selection signals for the various BRs and defense signaling pathways, which affect plant growth, development, and viability (Table 1). The 34 GO terms were involved in the selection, of which GO:0016132 (Brassinosteroid biosynthetic process) and GO:0042742 (Defense response to bacterium) were confirmed as major GO terms (Supplementary Fig. S8a and b). Among their 83 candidate genes, Glyma.16g170700, Glyma.16g210300, and Glyma.18g226500 genes (associated with the immune and defense responses to pathogens and insects) exhibited traces of selection process with long-range haplotypes and high LD peaks. Also, Glyma.08g323200 (associated with disease resistance) showed a trace of the selective sweep with hitchhiking event in the 44,174,470–44,174,678 bp region (Fig. 3C and Additional File 5). In line with our goal of revealing useful subgroups that can be utilized and referenced in future breeding studies and programs, this study statistically presented the adaptive characteristics of 4 soybean subgroups together with their associated candidate genes. Given our findings, we propose that the LR-1 subgroup could be a potential group with genetic material capable of coping with evolving SCN species, and that the IC-1 subgroup could be used for various breeding programs aimed at enhancing growth, development, and viability of soybeans. Additionally, the findings for the LR-2 and IC-2 subgroups would provide additional information on available donor parents to breeders seeking to increase SW, together with targeted genomic regions for candidate genes.

The article "Dissection of soybean populations according to selection signatures based on whole-genome sequences" was retracted in 2021. Reasons: an official misconduct investigation; misconduct by an author; concerns about the data.

In this study, our findings have several limitations. First, group variability might be implied among subgroups in each group. According to our hypothesis that the selection, adaptation, and bottleneck events have caused population stratification along with genomic difference, we classified each WT, LR, and IC group into 3, 2, and 2 subgroups based on the various population analyses. Each subgroup was maximized for both genomic similarity among accessions and genomic diversity between subgroups; however, this classification approach might have involved some variability problems for subgroups in which some accessions belonging to the boundaries between subgroups could be assigned to the other subgroup. To ensure the validity of our subgrouping, we utilized the WT group as a reference criterion of classification, and through its 3 subgroups classified according to China, Korea, and Japan origins, we indirectly confirmed that all subgroups have minimal subgroup variability together with their own genomic characteristics. Second, adaptive characteristics for 4 subgroups have been confirmed but not validated by biological experiments. To minimize this limitation, we used rigorous statistical approaches and conservative cut-offs in terms of genome analysis. We pairwise compared each subgroup with the other 3 subgroups and, for each comparison, regarded only genes belonging to the top 1% of the XP-CLR scores as candidate genes. Then, for each subgroup, we considered commonly detected candidate genes for all 3 other subgroups as the final candidate gene set representing each subgroup, in order to avoid all possible false-positive selection signals. Based on GSEA of these 4 gene sets, we derived the unique adaptive characteristics of each subgroup and presented some candidate genes relevant to their adaptive characteristics, together with genomic regions strongly affected by the selection pressures. Despite these efforts, our results still require further experimental validation, but the identified candidate genes and their focused genomic regions will be helpful in future experimental research aimed at utilizing the specific adaptive characteristics of each subgroup.

The article "Dissection of soybean populations according to selection signatures based on whole-genome sequences" was retracted in 2021. Reasons: an official misconduct investigation; misconduct by an author; concerns about the data.

### Potential implications

The genomic research carried out herein dissected the soybean population along population structures and revealed selection signatures within subpopulations, together with candidate genes. Although our findings for their adaptive characteristics are presented in the absence of biological validation, they provide not only targeted genomic regions to sequencing-based molecular breeding and marker-assisted breeding programs trying to use our hypotheses, but also present new options to breeders seeking donor parents to improve soybean populations. Additionally, our genomic resources that have been deposited in the public database can contribute useful data to other researchers.

## Methods

### Plant materials, sample preparation, and phenotypic evaluation

To construct a sample set for re-sequencing, we used genotype information of 4,234 soybean accessions comprising 2,824 CT, 1,360 WT, and 50 hybrid-type accessions collected from China, Korea, Japan, Russia, the USA, and other countries (Supplementary Fig. S1a and b). The 4,234 accession collection was developed through co-operation between our team and the Rural Development Administration (RDA, Jeonju, Korea) [29], and was genotyped using the 180 K Axiom^®^ SoyaSNP array, which our team also developed in 2016 [106]. The genotyped data are available [107]. From the 4,234 accessions, 245 core accessions were selected using the 0.95 coverage and 0.01 delta options within GenoCore software [108]. The core set comprised 112 WT and 133 CT (79 LR and 54 IC) soybean accessions and reflected ∼95% of the genotype frequency and diversity of the 4,234 accessions (Supplementary Table S1). Phenotypic evaluation was conducted on the CT group, and seeds of the 91 CT accessions (except for 42 CT accessions) were secured from the National Agrobiodiversity Center in the RDA. The seeds were sown in the experimental field at the National Institute of Crop Science (NICS, Jeonju, Korea) (35 50.445 N, 127 2.711 E) and grown during Korea's normal soybean-growing season, June to October, in 2016. Before planting, appropriate pesticides were used to control insects and weeds in the field and 40–70-60 kg/ha of N-P_2_O_5_-K_2_O was applied according to soil test recommendations. The planting arrangement was 70 × 15 cm per plot, and 3 replicates from each accession were planted for phenotypic measurement. The soil type was clay-loam, and the average monthly temperatures were 22.5°C, 25.8°C, 26.2°C, 21.5°C, and 15.0°C during June to October. Field management, including fertilizer application, irrigation, and pest control, followed the standard protocol for the normal agricultural practice of the RDA [109]. After harvesting, the soybean plants were dried in natural conditions and then threshed. When seed desiccation was complete, 100 normal seeds were randomly selected from each replicate of each accession and weighed. Average 100-SW for each accession was determined as the average of the 3 replicate values. The raw values of 100-SW of the 91 CT accessions are summarized in Additional File 2, and their distribution is shown in Fig. 5.

The article "Dissection of soybean populations according to selection signatures based on whole-genome sequences" was retracted in 2021. Reasons: an official misconduct investigation; misconduct by an author; concerns about the data.

### Genomic DNA extraction, re-sequencing, and data description

Seed from each of the 245 accessions was obtained from the National Agrobiodiversity Center (RDA, Jeonju, Korea) and germinated in pots sited in a dark growth chamber at 25°C. After the primary leaves germinated, all etiolated shoots except cotyledons were collected and genomic DNAs were extracted using the cetyl trimethylammonium bromide method. Among the extracted DNAs of the 245 accessions, 208 and 37 accessions were sequenced using Illumina NextSeq 500 and HiSeq 2000 platforms, respectively (Additional File 2). For NextSeq sequencing, sample libraries of 550 bp size were prepared using a TruSeq DNA PCR-Free Library Prep (Illumina, San Diego, CA) as follows. Genomic DNA (3 µg) was fragmented to 300–500 bp in size using a Covaris M220 sonicator (Covaris, Woburn, MA). The fragmented DNAs were then end-repaired by trimming 3ʹ overhangs and filling the 5ʹ overhangs, and size selected to remove large and small DNA fragments using Sample Purification Beads. An “A” nucleotide was added to the 3ʹ ends of the refined fragments to prevent fragments becoming ligated to one another, after which Illumina identifier indexes were ligated to the fragments of each sample. Prepared libraries were quantified using a KAPA Library Quantification Kit (Kapa Biosystems, Wilmington, MA) with a StepOnePlus Real-Time PCR System (Life Technologies, Carlsbad, CA). Size distributions were identified using Agilent 2100 Bioanalyzer Instruments (Agilent Technologies, Santa Clara, CA), and samples were then normalized and pooled into a single tube. Next, the pooled libraries were denatured and diluted to a final concentration of 1.9 pM following the Illumina NextSeq Denature and Dilution protocol with a 1% PhiX DNA spike for quality sequencing control. Finally, the pooled libraries were loaded onto 35 flow cells containing 4 lanes (∼6 accessions per flow cell) and sequenced as ∼151-bp paired-end reads with an average coverage of 15× (corresponding to 15  Gb per accession) on the Illumina NextSeq 500 sequencer with NextSeq 500 High Output v2 Kit (300 cycles) (Illumina). The binary-base-call format files generated from the sequencing were converted and demultiplexed into sequence files with data format of FastQ using Illumina Base Calling program bcl2fastq2 software v2.18. For HiSeq sequencing, 3 µg of genomic DNA was sheared to 300–500 bp fragment sizes using a Covaris LE220 focal acoustic device (Covaris), with default settings, and size selected using solid-phase reversible immobilization beads (Beckman Coulter). The size-selected fragments were then end-repaired, A-tailed, and ligated to Illumina sequencing adaptors containing a unique molecular index barcode for each sample library, using a KAPA-Illumina library creation kit (KAPA Biosystems). Then, the prepared libraries were quantified using the KAPA Biosystem next-generation sequencing library qPCR kit (KAPA Biosystems) with a Roche LightCycler 480 real-time PCR instrument. The quantified libraries were multiplexed with other sample libraries, and the library pools were clustered onto 6 flow cells containing 8 lanes through an Illumina cBot instrument with TruSeq PE Cluster Kit v3-cBot-HS (Illumina) (∼6 accessions per flow cell). The clustered flow cells were sequenced as ∼101-bp paired-end reads with an average coverage of 15× (corresponding to 15 Gb per accession) on the HiSeq 2000 sequencer using the TruSeq SBS sequencing Kit V3–HS (Illumina). The raw files generated from the sequencing were then converted and demultiplexed to sequence files with data format of FastQ using Illumina Base Calling programs bcl2fastq2 software v2.18.

The article "Dissection of soybean populations according to selection signatures based on whole-genome sequences" was retracted in 2021. Reasons: an official misconduct investigation; misconduct by an author; concerns about the data.

During the sequencing processes, Pureun accession (NextSeq 500) and Sowon, Hwangkeum, PI507822, PI424002, PI518282, and PI378691 accessions (HiSeq 2000) were sequenced a second time owing to low sequencing depth in the initial run. After sequencing, ∼23.18 billion reads (with 3,500 Gb) and 8.12 billion reads (with 818 Gb) were obtained in the FastQ files of 208 and 37 accessions generated from the NextSeq 500 and HiSeq 2000, respectively (Additional File 2). The averages of raw sequencing depth were ∼17× in the 208 accessions and 23× in the 37 accessions on the basis of the Wm82.a2.v1 reference gnome (949.74 Mb). The FastQ files for all accessions were deposited in the European Nucleotide Archive (ENA) under accession number PRJEB31453, and the detail information for each accession is provided in Additional File 2 (ENA sample ID, sequencer name, read length, FastQ file name, md5 checksum value, the number of reads, and the number of base pairs).

The article "Dissection of soybean populations according to selection signatures based on whole-genome sequences" was retracted in 2021. Reasons: an official misconduct investigation; misconduct by an author; concerns about the data.

### Data processing and variant calling

A per-base sequence quality check of raw FastQ files from 245 soybean accessions was conducted using FastQC v0.11.8 [110], and low-quality sequences were controlled using NGSQCToolkit v2.3.3 [111] (Additional File 2). The refined reads were mapped to a reference genome: *G. max*, Wm82.a2.v1 [30], using BWA v0.7.17 [112]. The chloroplast and mitochondrial genomes were excluded from this mapping step. The mapped files were sorted into the genomic coordinates of the Wm82.a2.v1 genome using the “AddOrReplaceReadGroup” option within Picard software v2.0.1, and potential PCR duplicates were eliminated using the “MarkDuplicates” option within the same software [113] (Additional File 2). To correct misalignments resulting from indels, the “RealignerTargetCreator” and “IndelRealigner” options within Genome Analysis Toolkit v3.7 (GATK) were applied [114]. Then, gVCF files for the 245 samples were generated using the GATK “HaplotypeCaller” option. The 245 gVCF files, called from all base sites of the reference genome, were combined into a single gVCF file using the GATK “CombineGVCFs” option and then converted to a single VCF file using the GATK “GenotypeVCFs” option. To exclude false-positive variants as much as possible, the GATK “Variant Filtration” and “Select Variants” arguments were adopted with the following options: (i) quality score by depth < 3.0; (ii) Phred-scale quality score < 30.0; (iii) mapping quality score < 30.0; (iv) genotype quality score < 10.0; (v) depth of coverage across all samples < 7.0; (vi) Phred-scale *P*-value score of the Fisher exact test for strand bias > 30.0; (vii) Rank-sum test for bias of relative positions of the reference and alternative alleles ≤ 2.0; and (viii) rank-sum test for mapping quality of the reference and alternative reads ≤ 2.0. Additionally, variants with a missing genotype rate of >15% were filtered to enable the use of comparatively common variants. After the strict quality filtering processes, the variants were separated into indel and SNP variants, and bi-allelic SNPs were extracted. For multi-allelic SNPs, an allele with the highest allele frequency was maintained as the only allele representing the corresponding SNPs, in order to reflect as many bi-allelic SNPs as possible covering all 245 soybean accessions. Haplotype phasing and imputation were then conducted to the bi-allelic SNPs using BEAGLE v4.1 [115], and bi-allelic SNPs with MAF > 1% were obtained (Supplementary Table S2). To identify variant distribution, SNP and indel variants of each group were detected in the same way, and their bi-allelic SNPs with MAF > 1% were obtained (Supplementary Table S3). At this time, multi-allelic SNPs were excluded for accurate comparisons between bi-allelic SNPs of each group. After that, functional effects of these bi-allelic SNPs on genomic regions were annotated through SnpEff v4.3 [116] using the Wm82.a2.v1 gene set (Supplementary Table S4).

The article "Dissection of soybean populations according to selection signatures based on whole-genome sequences" was retracted in 2021. Reasons: an official misconduct investigation; misconduct by an author; concerns about the data.

### Genomic statistics for populations

F of each sample was calculated using VCFtools v4.2 [117], and the F of each subgroup was obtained by averaging the F values of all samples belonging to each subgroup (Supplementary Table S5). π was calculated by sliding the genome to 50 kb, with a window size of 100 kb, using the same software. LD was calculated using Plink v1.90b [118] and measured as an adjusted *r*^2^ statistic. The mean values of all pairwise LDs within 30, 50, 100, and 500 kb regions are summarized in Supplementary Table S5, and the degree of LD decay up to 500 kb is provided in Fig. 2E and Supplementary Fig. S2.

### Genomic relationship and population structure

Fst [119] for all groups and subgroups was calculated in a pairwise manner by sliding the genome to 50 kb, with a window size of 100 kb, using VCFtools (Supplementary Table S6). The phylogenetic tree was reconstructed using RAxML v.8.2 [120], a software for inferring phylogenetic trees using a maximum likelihood approach based on sequence alignments of samples, and evaluated by the bootstrap using 1,000 replicates. Then, the reconstructed tree was visualized as a midpoint root through FigTree v1.4.3 [121] (Fig. 2A). Structure analysis was performed using FAST-STRUCTURE v1.0 [122], which uses a variational Bayesian framework for posterior inference (Fig. 2B). Genetic clusters were calculated from K = 2 to K = 5, as a 1.0 × 10^−7^ convergence criterion with 10× cross-validation. PC analysis was conducted by applying singular value decomposition to the distance matrix derived from the Kimura 2-parameter model [123], and this was displayed by PC1, PC2, and PC3 (Fig. 2C and D and Supplementary Fig. S3a–d). A maximum likelihood tree, which provides a population relationship with gene flow and genetic drift, was reconstructed using TreeMix v1.12 [124]. The whole WT group was used as 1 root group in order to focus more on interactions among the CT subgroups while minimizing the standard error because 2 subgroups in the WT group were small in sample size. Number of gene flows was set at 3, and block size for inferring a covariance matrix was 400 kb, taking into consideration the LD values (Supplementary Fig. S4). Scale bar represents the standard error of the tree estimated from the 10× calculations (Fig. 2F).

### Selection signals and gene set enrichment analysis

Detection of selection signals was performed using the cross-population composite likelihood ratio test within XP-CLR v1.0 [36]. A 10-kb sliding window with 50-kb window size was adopted to scan the whole genome. A maximum of 2,500 SNPs was used to compare the composite likelihood score in each window, and pairs of SNPs with an LD > 0.95 were down-weighted to minimize dependence effects on the scores. Because of the absence of an entirely constructed genetic map, genetic positions were assumed to be equivalent to physical positions (1 Mb = 1 cm). Outlier regions within the top 1% of the empirical distribution of the raw scores were considered to be putative selection regions (Supplementary Figs S5 and S6a–l), and genes belonging to these regions were designated as candidate selected genes (Supplementary Fig. S7a–d). Genes that spanned >80% at either side of these regions were also included as candidate genes. All results of the analyses are provided in Additional File 3. To reveal the patterns of the adaptation process, GSEA was performed using the PANTHER v14 database [125]. This analysis was conducted on biological processes in the PANTHER GO-Slim database and, only in the case of GO terms that did not exist in the database, was performed in the PANTHER GO database. Candidate selected genes were clustered into GO terms with similar functions in *G. max* through binomial testing. GO terms with a raw *P*-value < 0.05 and >3 candidate genes (except for GO terms where the total number of genes in the category was <3 genes) were considered to be statistically significant GO terms for selection signals (Table 1 and Additional File 4).

The article "Dissection of soybean populations according to selection signatures based on whole-genome sequences" was retracted in 2021. Reasons: an official misconduct investigation; misconduct by an author; concerns about the data.

To examine selection processes at gene level, the patterns of nucleotide diversity, haplotype diversity, and LD of the candidate selected genes were calculated using the methods presented by Hudson et al. [46], Nei [47], and Kelly [48] (Table 2, Figs 3A and B and 4A and B). Plots for the degree of haplotype sharing that indirectly present the selective sweep were generated using R [126] and were visualized by assigning major and minor alleles of each variant in a target gene as red and yellow, respectively (Figs 3A and B and 4A and B). Haplotype frequencies of a region containing 1 or 2 missense variants in a target gene were calculated by including 14 variants surrounding the missense variant as tag SNPs, and were computed using Plink v1.90b [118] (Figs 3C and D and 4C and D, and Additional File 5). The haplotype frequencies of each subgroup are shown to the right of the corresponding haplotype structures, below gene structure. Reference and alternative alleles (Alleles 1 and 2) are presented in green and yellow, and missense variants are marked a light yellow. Owing to illustration size constraints, only the top 2 haplotype frequencies are displayed for each subgroup. Information regarding all haplotype frequencies is provided in Additional File 5. All calculations used the 19,853,829 bi-allelic SNPs without MAF filtering to consider fixed SNP variants due to selection process.

The article "Dissection of soybean populations according to selection signatures based on whole-genome sequences" was retracted in 2021. Reasons: an official misconduct investigation; misconduct by an author; concerns about the data.

## Availability of Supporting Data and Materials

The 245 soybean whole genomes are publicly available in the ENA and the European Variation Archive under accession numbers PRJEB31453 and PRJEB35532. The accession IDs and sample IDs for all samples are provided in Additional File 2. Supporting data, including VCF files, are also available via the *GigaScience* database GigaDB [127].

## Additional Files

Additional File 1: Supplemental Table S1. Origins of the 112 wild and 133 cultivar soybeans.

Supplemental Table S2. Number of variants detected along the 20 chromsomes in entire soybean samples.

Supplemental Table S3. Number of variants detected in each group and subgroup.

Supplemental Table S4. Number of bi-allelic SNPs with functional effects on the genome and protein regions in each group and subgroup.

Supplemental Table S5. Genomic diversity (π), inbreeding coefficient (F), and average linkage disequilibrium (LD) values for each group and subgroup.

Supplemental Table S6. Mean Fst values for each group and subgroup.

Supplemental Figure S1. PC analysis plot of 4,234 soybean samples containing our CT and WT soybean samples. The gray circles represent 4,234 soybean samples. **a**, PC analysis plot for 2,824 CT samples including our 133 CT samples. **b**, PC analysis plot for 1,360 WT samples including our 112 WT samples. Among the 4,234 samples, 50 CT samples close to hybrid were excluded from this study.

Supplemental Figure S2. Extent of LD decay for IC, LR, and WT groups.

Supplemental Figure S3. PC analysis for all groups and cultivar groups. **a**,PC analysis plot for all groups, visualized using PC2 and PC3 of Figure 2C. **b**, Scree plot for all groups. **c**, PC analysis plot for only cultivar groups, visualized using PC2 and PC3 of Figure 2D. **d**, Scree plot for only cultivar groups.

Supplemental Figure S4. Residual matrix of the maximum-likelihood tree shown in Figure 2F. Closeness of the residual value of a group pair to 0.2 or -0.2 indicates a more closely related group pair that can be a candidate for a gene flow event.

Supplemental Figure S5. Distribution of XP-CLR raw scores. Each plot contains the names of the subgroups that were compared in the XP-CLR calculations.

Supplemental Figure S6. Manhattan plots showing the results of selection analyses conducted using XP-CLR. Each of the four subgroups was compared pairwise with the other three subgroups. **a, b, c**, Comparison of IC-1 with IC-2, LR-1, and LR-2. **d, e, f**, Comparison of IC-2 with IC-1, LR-1, and LR-2. **g, h, i**, Comparison of LR-1 with IC-1, IC-2, and LR-2. **j, k, l**, Comparison of LR-2 with IC-1, IC-2, and LR-1. The blue and red dotted lines represent the top 0.5% and 1% cutoffs of the empirical distributions of XP-CLR results, respectively.

The article "Dissection of soybean populations according to selection signatures based on whole-genome sequences" was retracted in 2021. Reasons: an official misconduct investigation; misconduct by an author; concerns about the data.

Supplemental Figure S7. Number of candidate genes for each subgroup pair detected by XP-CLR analyses. **a–d**, In the top 1% of the empirical distributions of XP-CLR results (Figures S5 and S6), IC-1, IC-2, LR-1, and LR-2 had 422, 235, 454, and 258 candidate genes detected in common, respectively (see Additional file 3 for all candidate genes of XP-CLR analysis results).

Supplemental Figure S8. GO term relationship plots for biological functions of GO:0016132 and GO:0042742 among GO terms in which IC-1's candidate genes are significantly enriched. **a**, GO:0016132 (Brassinosteroid biosynthetic process) is directly associated with IC-1’s 15 other GO terms. **b**, GO:0042742 (The defense response to bacterium) is directly related to IC-1’s eight other GO terms. These GO term relationship plots were generated through the QuickGO database. Statistically significant GO terms identified in the GSEA are outlined in red (see Additional file 4 for all GO terms of GSEA results).

Supplemental Figure S9. GO term relationship plot for biological functions of GO:0009793 among the GO terms in which IC-2's candidate genes are significantly enriched. The GO:0009793 (The embryo development ending in seed) is directly associated with the IC-2’s 14 other GO terms. The GO term relationship plot was generated through the QuickGO database. Statistically significant GO terms identified in the GSEA are outlined in red (see Additional file 4 for all GO terms of GSEA results).

Supplemental Figure S10. GO term relationship plots for biological functions of GO:0009624, GO:0045087, and GO:0051172 among the GO terms in which LR-1's candidate genes are significantly enriched. **a**, GO:0009624 (Response to nematode) is directly connected with LR-1’s six other GO terms. **b**, GO:0045087 (Innate immune response) is directly associated with LR-1’s 10 other GO terms. **c**, GO:0051172 (Negative regulation of nitrogen) is directly related to LR-1’s six other GO terms. These GO term relationship plots were generated through the QuickGO database. Statistically significant GO terms identified in the GSEA are outlined in red (see Additional file 4 for all GO terms of GSEA results).

Supplemental Figure S11. GO term relationship plots for biological functions of GO:0010431, GO:0010029, and GO:0043043 among the GO terms in which LR-2's candidate genes are significantly enriched. **a**, GO:0010431 (Seed maturation) is directly associated with LR-2’s 10 other GO terms. **b**,GO:0010029 (Regulation of seed germination) is directly connected with LR-2’s eight other GO terms. **c**, GO:0043043 (Peptide biosynthetic process) is directly related to LR-2’s 14 other GO terms. These GO term relationship plots were generated through the QuickGO database. Statistically significant GO terms identified in the GSEA are outlined in red (see Additional file 4 for all GO terms of GSEA results).

The article "Dissection of soybean populations according to selection signatures based on whole-genome sequences" was retracted in 2021. Reasons: an official misconduct investigation; misconduct by an author; concerns about the data.

Supplemental Figure S12. Selection signals for IC-1 in Glyma.16g210300. **a, b, c**,Patterns of nucleotide diversity, haplotype diversity and linkage disequilibrium for IC-1, IC-2, LR-1, LR-2, WT-1, WT-2, and WT-3, in the gene region located at bp 36,943,073–36,948,828 on chromosome 16. The IC-1 subgroup is depicted in dark green.

Supplemental Figure S13. Selection signals for IC-1 in Glyma.16g170700 and Glyma.18g226500. **a, b**, Patterns of nucleotide diversity, haplotype diversity, and linkage disequilibrium (top) and the degree of haplotype sharing among all subgroups (bottom) in Glyma.16g170700 and Glyma.18g226500, respectively. Glyma.16g170700 is located at bp 33,101,084–33,105,462 on chromosome 16, and Glyma.18g226500 is located at bp 51,507,715–51,550,797 on chromosome 18. All seven-subgroup lines are displayed for the three characteristics patterns. Haplotype sharing plots are displayed for all variants in the entire regions of two genes, and the major and minor alleles of each variant are shown in red and yellow, respectively. The IC-1 subgroup is depicted in dark green.

Supplemental Figure S14. Selection signals for IC-2 in Glyma.03g144400. **a, b, c**, Patterns of nucleotide diversity, haplotype diversity and linkage disequilibrium for IC-1, IC-2, LR-1, LR-2, WT-1, WT-2, and WT-3, in the gene region located at bp 36,004,707–36,005,955 on chromosome 3. The IC-2 subgroup is depicted in pale green.

Supplemental Figure S15. Selection signals for IC-2 in Glyma.03g022900. **a, b, c**, Patterns of nucleotide diversity, haplotype diversity and linkage disequilibrium for IC-1, IC-2, LR-1, LR-2, WT-1, WT-2, and WT-3, in the gene region located at bp 2,409,690–2,420,328 on chromosome 3. The IC-2 subgroup is depicted in pale green.

Supplemental Figure S16. Selection signals for LR-2 in Glyma.12g181400. **a, b, c**, Patterns of nucleotide diversity, haplotype diversity and linkage disequilibrium for IC-1, IC-2, LR-1, LR-2, WT-1, WT-2, and WT-3, in the gene region located at bp 34,193,664–34,197,110 on chromosome 12. The LR-2 subgroup is depicted in navy blue.

The article "Dissection of soybean populations according to selection signatures based on whole-genome sequences" was retracted in 2021. Reasons: an official misconduct investigation; misconduct by an author; concerns about the data.

Supplemental Figure S17. Selection signals for LR-2 in the Glyma.12g028300-Glyma.12g028400 genes. Patterns of nucleotide diversity, haplotype diversity, and linkage disequilibrium (top) and the degree of haplotype sharing among all subgroups (bottom), in the two genes located at bp 2,111,211-2,128,944 on chromosome 12. All seven-subgroup lines are displayed for the three characteristic patterns. Haplotype sharing plot is displayed for all variants in the entire regions of two genes, and the major and minor alleles of each variant are marked in red and yellow, respectively. The LR-2 subgroup is depicted in navy blue.

Supplemental Figure S18. Selection signals for LR-1 in Glyma.03g051100. **a, b, c**,Patterns of nucleotide diversity, haplotype diversity and linkage disequilibrium for IC-1, IC-2, LR-1, LR-2, WT-1, WT-2, and WT-3, in the gene region located at bp 6,684,296–6,686,809 on chromosome 3. The LR-1 subgroup is depicted in light blue.

Supplemental Figure S19. Selection signals for LR-1 in Glyma.14g047900. Patterns of nucleotide diversity, haplotype diversity, and linkage disequilibrium (top) and the degree of haplotype sharing among all subgroups (bottom), in the gene located at bp 3,674,123-3,677,641 on chromosome 14. All seven-subgroup lines are displayed for the three characteristic patterns. Haplotype sharing plot is displayed for all variants in the entire region of this gene, and the major and minor alleles of each variant are marked in red and yellow, respectively. The LR-1 subgroup is depicted in light blue.

Additional File 2: Summary of the samples' origins, phenotype, re-sequencing information, and mapping statistics.

Additional File 3: Summary of the results of the XP-CLR analyses.

Additional File 4: Summary of the results of the gene set enrichment analyses.

Additional File 5: Summary of the 5 missense variants and their surrounding haplotype frequencies.

giz151_GIGA-D-19-00118_Original_Submission

giz151_GIGA-D-19-00118_Revision_1

giz151_GIGA-D-19-00118_Revision_2

giz151_GIGA-D-19-00118_Revision_3

giz151_Response_to_Reviewer_Comments_Original_Submission

giz151_Response_to_Reviewer_Comments_Revision_1

giz151_Response_to_Reviewer_Comments_Revision_2

giz151_Reviewer_1_Report_Original_Submission Anne V Brown, Ph.D -- 5/21/2019 Reviewed

giz151_Reviewer_1_Report_Revision_1 Anne V Brown, Ph.D -- 9/6/2019 Reviewed

giz151_Reviewer_1_Report_Revision_2 Anne V Brown, Ph.D -- 11/12/2019 Reviewed

giz151_Reviewer_2_Report_Original_Submission Jason Gillman -- 5/30/2019 Reviewed

giz151_Reviewer_2_Report_Revision_1 Jason Gillman -- 9/6/2019 Reviewed

giz151_Supplemental_Files

## Abbreviations

bp: base pairs; BR: Brassinosteroids; BWA: Burrows-Wheeler Aligner; CLR: composite likelihood ratio; CT: cultivar-type; ENA: European Nucleotide Archive; F: inbreeding coefficient; Fst: fixation index value; GATK: Genome Analysis Toolkit; Gb: gigabase pairs; GO: Gene Ontology; GSEA: gene-set enrichment analysis; HG: *Heterodera glycines*; IC: improvement cultivar; indel: insertion/deletion polymorphism; kb: kilobase pairs; LD: linkage disequilibrium; LR: landrace cultivar; MAF: minor allele frequency; Mb: megabase pairs; PC: principal component; π: genomic diversity; QTL: quantitative trait locus; RDA: Rural Development Administration; SCN: soybean cyst nematode; SNP: single-nucleotide polymorphism; SW: seed weight; Wm82.a2.v1: Williams 82 assembly 2 annotation version 1; WT: wild type; XP-CLR: cross-population composite likelihood ratio.

The article "Dissection of soybean populations according to selection signatures based on whole-genome sequences" was retracted in 2021. Reasons: an official misconduct investigation; misconduct by an author; concerns about the data.

## Competing interests

The authors declare that they have no competing interests.

## Funding

This study was supported by grants from KRIBB Initiative program, National Research Foundation of Korea (NRF-2014M3C9A3064552), and Rural Development Administration of Korea (PJ01313201).

## Authors' Contributions

N.K. designed and supervised this project. J.-Y.K. and S.J. performed data analysis and wrote the manuscript. K.H.K. and W.-J.L. assisted in data analysis and interpretation. H.-Y.L. supported figure preparation and literature search. N.J. conducted the phenotypic investigation. J.-K.M. collected samples, extracted genomic DNA, and re-sequenced the samples.
